RETRACTED

# Investigation of the Clinical Application Value of HR-HPV DNA Combined with Liquid Based Cytology in Colposcopy of Cervical Cancer

**DOI:** 10.1155/2022/5054507

**Published:** 2022-08-29

**Authors:** Ying Zhou

**Affiliations:** Obstetrics and Gynecology Department, The First Affiliated Hospital of Xiamen University, Xiamen 361000, China

## Abstract

In order to investigate the clinical application value of HR-HPV DNA combined with liquid-based cytology in colposcopy of cervical cancer, a retrospective analysis is performed on 428 patients who underwent a cervical pathological examination in our hospital from May 2020 to December 2021. The pathological biopsy results are used as the gold standard to determine whether cervical lesions occurred in patients, and patients with positive gold standard results are included in the study group. The positive rates of liquid-based cytology and HR-HPV DNA are observed and recorded, and the patients with negative gold standard results are used as the control group. The positive rate of HR-HPV DNA and liquid-based cytology will increase with the aggravation of pathological results. The ROC curve shows that HR-HPV DNA combined with liquid-based cytology has high diagnostic efficiency in colposcopy of cervical lesions. It is clearly evident that both liquid-based cytology and HR-HPV DNA tests have certain advantages in the screening of cervical lesions, and the combined detection can further improve the screening value of cervical lesions.

## 1. Introduction

Cervical cancer is one of the most common gynecological tumors. Cervical intraepithelial neoplasia develops over a long period of time and reverses precancerous lesions, and finally forms cervical cancer. Therefore, early diagnosis and treatment of cervical lesions can effectively prevent the further development of cervical cancer and improve the prognosis of patients [1, 2]. A Pap smear was a commonly used cervical cytological examination method in clinical practice in the past. However, with the continuous improvement of medical technology, this method is no longer applicable to modern clinical practice. As a new cytological smear method, the cervical cells prepared by liquid-based cytology have a clear structure and can improve the detection sensitivity. Some related studies also show that it has a good diagnostic effect [3]. However, some scholars have proposed that cytology alone cannot completely screen cervical lesions. They emphasized that human papillomavirus (HPV), as one of the risk factors for cervical lesions, almost exists in most patients with cervical lesions. Although some HPV infections can naturally subside under the action of the human immune system, some HPV infections combined with atypical hyperplasia may lead to varying degrees of cervical lesions [4]. As a morphological examination method of cervical lesions, colposcopy combined with cytology and pathology can effectively improve diagnostic efficiency and play an important role in treatment. However, some patients with relatively narrow cervices were not fully exposed [5, 6]. Therefore, the location of the lesion may lead to missed diagnosis and misdiagnosis. Based on the advantages and disadvantages of the above cervical lesion detection methods, liquid-based cytology and HR-HPV DNA detection on patients of our hospital for cervical lesion screening from May 2020 to December 2021 was conducted to explore the clinical value of liquid-based cytology and HR-HPV DNA detection in the early diagnosis of cervical lesions and to provide a theoretical basis for the treatment of such patients in the future.

RETRACTED

The rest of the study is organized as follows: section 2 discusses related work, and section 3 presents the test methods and indicators.  Section 4 describes the results and analysis. In section 5, the conclusions are presented.

## 2. Related Work

As one of the common female reproductive tract tumors, cervical cancer is often caused by cervical HPV infection caused by bad living habits. According to the statistical data of WHO, the incidence rate of cervical cancer is increasing year by year, and the incidence group is gradually getting younger [7]. There are about 500,000 cases of cervical cancer worldwide every year, accounting for about 30% of all new cases. In particular, patients with a history of multiple pregnancies or uterine cavity surgery have a higher probability of cervical lesions [8]. Although it has a high incidence rate, the incidence of cervical cancer is a slow development process from quantitative change to qualitative change. If treated in time in the early diagnosis of cervical lesions, the prognosis of patients with cervical lesions can be greatly improved, which is of great significance in preventing the development of cervical cancer [9]. At present, in clinical practice, microscopic examination is often used to diagnose cervical cancer and precancerous lesions through vaginal screening. Studying the iodine staining of cervical tissue and colposcopy observation can evaluate the risk of cervical lesions and provide the basis for clinical treatment. Due to the long time and high cost of examination and operation, as well as the cervical bleeding caused by improper operation during the examination, the patient's compliance and acceptance of the test are relatively low [10]. Therefore, it is urgent to find a reliable and convenient diagnostic method in clinical examination to realize the early diagnosis of cervical lesions.

RETRACTED

With the continuous development of society, the level of medical technology is also improving. Liquid-based cytology has gradually replaced the traditional Pap smear in specimen collection and specimen preparation technology, and according to some studies, the positive detection rate of liquid-based cytology in squamous epithelial lesions and cervical cancer can reach 93% and 100%, respectively. However, the positive detection rates of traditional Pap smears in the above two cervical lesions are 77.80% and 90.90%, respectively [11, 12]. The results of this study showed that the positive rate of liquid-based cytology test results increased with the increase of pathological grade. Liang et al. [13] indicated that some patients with ASCUS detected by liquid-based cytology may be diagnosed with benign lesions or potential malignant changes, which cannot be clearly classified and diagnosed but can only be suggested for the presence of lesions, which is quite different from the gold standard of pathological biopsy under colposcopy. Therefore, cytological test results alone cannot be used as pathological criteria in clinical practice. HPV infection is one of the main factors of cervical cancer and precancerous lesions. Most studies have proved that only persistent high-risk HPV infection can cause cervical cancer. Most women only carry the virus, but it will not develop. Relevant statistics show that with the aggravation of cervical lesions, the HPV infection rate will also increase. Therefore, HR-HPV DNA testing is one of the important methods for cervical cancer screening in clinical practice [14, 15]. The positive rate of the HR-HPV DNA test increased with the increase of pathological grade, indicating that HPV infection is closely related to the occurrence of cervical lesions. However, the medical community has not reached a consensus on the connection between the degree of cervical lesions and virus load. Thus, genotyping is performed only on HR-HPV DNA testing and is classified as high-risk and low-risk. The above results all illustrate the same view, that is, if the patient's HPV test result is positive, it cannot be completely determined whether the patient has cervical lesions. Only patients with the HPV virus and the persistence of HPV can develop cervical lesions. If the liquid-based cytology test is negative, it cannot indicate that there is no cervical lesion. It indicates that the false negative results of liquid-based cytology tests are caused by various factors such as equipment and doctors' operations [16, 17].

Based on the advantages and disadvantages of the above liquid-based cytology and HR-HPV DNA tests, this study evaluated the value of their early diagnosis of cervical lesions under colposcopy by combining the two tests and drawing ROC curves. Results show that the liquid-based cytology joint HR—HPV DNA testing area under the curve is significantly higher than the single detection, illustrating the two means of joint detection as a screening of cervical cancer and precancerous lesions. Through accurate screening tests for biopsy under colposcopy clear objectives, for patients with cervical lesions can reduce the physical pain in the inspection process. For patients with cervical lesions, the diagnosis rate can be effectively improved, and corresponding treatment measures can be taken in the early stages to prevent the further development of the disease [18, 19].

RETRACTED

## 3. Test Methods and Indicators

### 3.1. General Information

A retrospective analysis was performed on 428 patients who underwent cervical pathology examination in our hospital from May 2020 to December 2021. All patients in both groups had completed liquid-based cytology and HR-HPV tests. The pathological biopsy results are used as the gold standard to determine whether cervical lesions occurred in patients. The mean age was (36.49 ± 6.32) years, the mean gestation was (1.29 ± 0.21) times from 0 to 3 times, and 312 (72.90%) of the patients had a birth history. Patients with negative gold standard results are used as a control group. All patients are forbidden to use vaginal cleaning drugs for vaginal irrigation within 3 days before examination and for sexual activity within 48 hours. Relevant examinations should be carried out during nonmenstrual periods, and lubricants should not be used during the examination. All patients enrolled in the study signed informed consent.

Inclusion criteria are as follows: (1) meet the clinical diagnostic criteria for cervical precancerous lesions; (2) complete clinical data and general information; (3) nonlactation, pregnancy, and menstruation; (4) no other gynecological inflammatory diseases.

Exclusion criteria are as follows: (1) suffering from mental diseases and unable to cooperate with researchers; (2) checking those who have had sex within 24 hours; (3) no sexual life history; (4) persons with severe organ and tissue dysfunction.

### 3.2. Methods

#### 3.2.1. HR HPV DNA Testing

13 high-risk HPV subtypes including HPV (16, 18, 31, 33, 35, 39, 45, 51, 52, 56, 58, 59, and 68) in cervical canal samples are detected by digene instruments and the hybrid capture (HC-2) method. HR-HPV DNA≥1.0 ng/L can be interpreted as a positive result, and the specific testing procedures are as follows:

**Step 1 .**

RETRACTED

Cracking. Specimen collection: On the basis that the patient had no vaginal irrigation for 3 days and had no sexual activity within 24 hours and was not hemorrhagic, a cervical sampler (manufacturer: Digene) is used to collect specimens and send them to the laboratory. Each test tube is marked and 5 drops of the indicator are added into the lysate to shake well. The negative control is added with 1000 *μ*l lysate, and the positive control and specimens are added with 500 *μ*L lysate, respectively. Mix well and then take a water bath at 65°C until each test tube appears purple. Replace gloves with an HC2 probe. Next, take out the tube holder, mix the tubes evenly, open the screw cover, and leave it at room temperature for about 15 min.

**Step 2 .**

Hybridization. Absorb 75 *μ*L of mixed and cracked control and all sample solution into each well. Absorb 25 *μ*L of prepared probe solution (probe) into a 96-well microplate; cover the cover and put it in the oscillator 1100 ± 100 rpm for mixing for 3 min; check that the liquid in all holes is yellow; put in HC2 constant temperature heater 65°C incubation for 60 min; remove cover immediately and leave for 5 minutes to cool.

**Step 3 .**

Capture. Transfer the liquid from each hole (100 *μ*L) to the capture hole, and cover the cover; the plate is placed in the HC2 oscillator (1100 ± 100 rpm) for 60 min; discard the liquid in the hole, and pat firmly on absorbent paper until dry.

**Step 4 .**

Reaction. Absorb 75 *μ*L DR1 solution (detection reagent1) into each hole, cover the cover plate at 20 to 25°C for 30 min, and the rinse solution (100 ml Ish buffer mixed with 2900 ml distilled water) is configured. Cover the board with absorbent paper, quickly turn over to discard the liquid, and vigorously slap the board on the paper until dry.

**Step 5 .**

Ishing plate. Ish at least 6 times (vertical to the bottom, there must be some momentum); pat the board vigorously on absorbent paper, and place it on the paper for 5 minutes until dry. Change gloves and wear a mask.

**Step 6 .**

Signal amplification and instrument interpretation. 75 *μ*L DR2 solution is added to each well and allowed to stand for 15 min in the dark condition at 20–25°C. DML200 is used to interpret the results.

#### 3.2.2. Liquid Based Cytology Detection

In the U.S. liquid-based cytology of Hologic company's production technology for the sample under a microscope in the cervix cytology diagnosis classification, specific steps are as follows: (1) *The Specimen Collection*. In patients with 3 d douching and asexual behavior within 24 h, and the period under the basis of the samples taken into the bottle containing cell preservation solution, and sent to test; (2) each sample consumable shall be marked separately, including sample preservation bottle, centrifugal tube, and glass slide; put the sample preservation bottle into the oscillator (single head/multiple heads), oscillate and mix the sample for 15 s (5 s can be increased or decreased), speed: 3000 rpm; (3) put the sample preservation bottle, centrifugal tube, and syringe into the PrepMate TM sample transfer rack. The storage bottle and the centrifugal tube must correspond correctly; (4) add 4 ml sample density separation solution to each empty centrifuge tube; (5) the slide holder shall be marked to ensure, that it is correctly corresponding to the sample transfer holder number; settling chamber; (6) run the automatic sample transfer machine, start the self-check first and put the sample transfer rack into the transfer machine; add or subtract the number of samples by pressing INC or DEC; (7) centrifuge at 200 g for the first gentle rotation centrifuge, selection procedure 1 centrifugal 2 min 15 s; (8) after centrifugation, use a suction pump to remove impurities such as blood and mucus from the upper layer of the centrifugal tube; (9) *Selection Procedure 2*: perform the second strong rotation centrifugation at 800 g for 10 min; (10) remove the excess impurities by gently pouring the excess liquid 180° down the centrifuge tube holder; (11) after fully oscillating the centrifugal tube rack for 15 s, put the centrifugal tube rack and the glass slide into the PrepStain TM production system to adjust the centrifugal tube rack and the glass slide rack. Check all the liquid levels of the dye and the label of the suction tube, place the dye tube, and run the PrepStain TM production system; (12) microscopically, the evaluation criteria are classified as inflammatory or normal (NIML), atypical squamous epithelial cells with little significance (ASCUS), high squamous cell neoplasia (ASC-H), low grade squamous intraepithelial lesion (LSIL), high squamous intraepithelial lesion (HSIL), squamous cell carcinoma (SCC), and low-grade squamous cell neoplasia (LSIL). ASCUS and the above lesions are interpreted as positive results.

RETRACTED

#### 3.2.3. Case Biopsy under Colposcopy

The colposcopic biopsy will enlarge the suspected cervical lesions. Add acetic acid or iodine solution to make the lesion clearer under the electron microscope. Thus, the pathological changes of the cervical epithelium can be observed. The specific procedures are as follows: (1) During the phase of specimen collection, 3–5% acetic acid and Lugo's iodine solution are applied to the cervical surface, respectively, and the color changes are observed. It should be noted that the patient had no vaginal irrigation for 3 days and had no sexual activity within 24 hours and is not in a menstrual period. Besides, pathological tissues are collected from suspicious parts by colposcopy and sent for examination. (2) Electron microscopy and diagnostic grading are performed under an electronic microscope, and cervical epithelial cells are classified into mild atypical hyperplasia (CIN I) according to the degree of cell variation; moderate atypical hyperplasia (CIN II); severe atypical hyperplasia and cervical carcinoma in situ (CIN III). Cervical cancer of CIN II or above is considered positive.

### 3.3. Observation Indicators

The observation indicators include: (1) gold standard results of pathological biopsy; (2) HR-HPV DNA test results and comparison with the gold standard; (3) liquid-based cytology detection results and comparison with the gold standard; (4) draw receiver operating characteristic (ROC) curve to evaluate the screening value of combined detection and single detection for early cervical lesions.

### 3.4. Statistical Processing

The SPSS 25.0 statistical software is used for data analysis. Enumeration data: described by sample number and percentage, compared by *X*^2^ test. To evaluate the ROC value of combined and single tests for screening early cervical lesions. *P* < 0.05 indicated a statistically significant difference.

## 4. Results and Analysis

### 4.1. Gold Standard Results of Pathological Biopsy

Pathological results showed that among the 428 patients, 124 cases (28.97%) are inflammatory reactions, 76 cases (17.76%) are CIN I, 110 cases (25.70%) are CIN II, 81 cases (18.93%) are CIN III, and 37 cases (8.64%) are cervical cancer. A total of 228 cases (53.27%) are pathologically positive, as shown in Table 1.

### 4.2. HR-HPV DNA Test Results and Comparison with Gold Standard

The positive rate of HR-HPV DNA increased with the aggravation of pathological results, and the positive rate of CIN (I, II, and III) and cervical cancer is significantly higher than that of inflammation, while the positive rate of CIN (II and III) and cervical cancer is significantly higher than that of CINI (all *P* < 0.05), as shown in Table 2. The mark “^*∗*^” indicates that compared with inflammation, ^*∗*^*P* < 0.05. The mark “^#^” means that compared with CIN I, ^#^*P* < 0.05.

### 4.3. Liquid Based Cytology Detection Results and Comparison with Gold Standard

The positive rate of CIN (I, II, and III) and cervical cancer is significantly higher than that of inflammation, and the positive rate of CIN III and cervical cancer is significantly higher than that of CIN I (all *P* < 0.05), as shown in Table 3. Besides, the different types of cervical lesions are detected by liquid-based cytology. Figures 1 and 2 demonstrate the comparison of ASCUS, ASC-H, and LSIL, and the comparison of HSIL and SCC, respectively.

RETRACTED

### 4.4. ROC Curve of the Diagnostic Efficacy of Combined Diagnosis and Single Diagnosis for Cervical Lesions under Colposcopy

The diagnostic efficacy is shown in Table 4. The ROC curve showed that the area under the ROC curve of combined detection is significantly higher than that of liquid-based cytology and HR-HPV DNA alone, indicating that combined detection had higher diagnostic efficacy for cervical lesions (*P* < 0.05), as shown in Figure 3.

## 5. Conclusions

In this study, the clinical application value of HR-HPV DNA combined with liquid-based cytology in colposcopy of cervical cancer is investigated. A retrospective analysis was performed on 428 patients who underwent a cervical pathological examination in our hospital from May 2020 to December 2021. The pathological biopsy results are used as the gold standard to determine whether cervical lesions occurred in patients, and patients with positive gold standard results are included in the study group. The positive rates of liquid-based cytology and HR-HPV DNA are observed and recorded, and the patients with negative gold standard results are used as the control group. The positive rate of HR-HPV DNA and liquid-based cytology will increase with the aggravation of pathological results. The ROC curve shows that HR-HPV DNA combined with liquid-based cytology has high diagnostic efficiency in colposcopy of cervical lesions. HR-HPV DNA combined with liquid-based cytology detection can improve the positive detection rate of cervical lesions under colposcopy, and reduce misdiagnosis and missed diagnosis by making up for their limitations and shortcomings. This study research results are of great significance in determining early cervical lesions and improving the prognosis of such patients.

## Figures and Tables

**Figure 1:** Comparison of ASCUS, ASC-H, and LSIL: (a) ASCUS; (b) ASC-H; and (c) LSIL.

**Figure 2:** Comparison of HSIL and SCC: (a) HSIL and (b) SCC.

**Figure 3:** ROC curve of the diagnostic efficacy of combined diagnosis and single diagnosis for cervical lesions under colposcopy.

**Table 1:** Pathological results.

	The total number of cases	Number	Ratio (%)
Inflammation	428	124	28.97
CIN I	428	76	17.76
CIN II	428	110	25.70
CIN III	428	81	18.93
Cervical cancer	428	37	8.64
Positive rate	428	228	53.27

**Table 2:** HR-HPV DNA test results and comparison with the gold standard.

	Number	HR-HPV DNA	
		Positive	Negative
Inflammation	124	15 (12.10%)	109 (87.90%)
CIN I	76	31 (40.79%)^*∗*^	45 (59.21%)
CIN II	110	69 (62.73%)^*∗*^^#^	41 (37.27%)
CIN III	81	74 (91.36%)^*∗*^^#^	7 (8.64%)
Cervical cancer	37	34 (91.89%)^*∗*^^#^	3 (8.11%)
Total	428	223 (52.10%)	205 (47.90%)

RETRACTED

**Table 3:** Liquid-based cytology detection results and comparison with the gold standard.

	Number	Liquid-based cytology						Positive rate
		NILM	ASCUS	ASC-H	LSIL	HSIL	SCC	
Inflammation	124	120	3	1	0	0	0	4 (3.23%)
CIN I	76	12	42	16	5	1	0	64 (84.21%)^*∗*^
CIN II	110	15	46	24	17	8	0	95 (86.36%)^*∗*^
CIN III	81	0	17	34	20	10	0	81 (100.00%)^*∗*^^#^
Cervical cancer	37	0	0	0	0	0	37	37 (100.00%)^*∗*^^#^
Total	428	147	108	74	52	9	25	268 (62.62%)

**Table 4:** Diagnostic performance table.

Index	95% CI	*P*	Sensitivity (%)	Specificity (%)	AUC
The joint detection	0.888–0.948	0.015	92.10	91.50	0.918
Liquid-based cytology	0.855–0.924	0.018	89.90	88.10	0.890
HR-HPV DNA	0.853–0.922	0.018	89.00	88.60	0.888

## Data Availability

The simulation experiment data used to support the findings of this study are available from the corresponding author upon request.
